# Social Norms about a Health Issue in Work Group Networks

**DOI:** 10.3390/ijerph120911621

**Published:** 2015-09-16

**Authors:** Lauren B. Frank

**Affiliations:** Department of Communication, Portland State University, Portland, OR 97201-0751, USA; E-Mail: lfrank@pdx.edu; Tel.: +1-503-725-3575; Fax: +1-503-725-5385

**Keywords:** social norms, small groups, social network analysis, cognitive social structure, H1N1 flu

## Abstract

The purpose of this study is to advance theorizing about how small groups understand health issues through the use of social network analysis. To achieve this goal, an adapted cognitive social structure examines group social norms around a specific health issue, H1N1 flu prevention. As predicted, individual’s attitudes, self-efficacy, and perceived social norms were each positively associated with behavioral intentions for at least one of the H1N1 health behaviors studied. Moreover, collective norms of the whole group were also associated with behavioral intentions, even after controlling for how individual group members perceive those norms. For members of work groups in which pairs were perceived to agree in their support for H1N1 vaccination, the effect of individually perceived group norms on behavioral intentions was stronger than for groups with less agreement.

## 1. Introduction

Calls to incorporate greater consideration of the social and cultural aspects of the health environment [1,2] have led to more nuanced theorizing about the role of social norms in the understanding of health decisions [3,4] and of social networks in influencing these social norms [5,6,7]. However, the theoretical recognition of the importance of social determinants to health has outpaced methodological tests of these determinants. By incorporating social network analytic techniques, the purpose of this study is to incorporate and empirically test how people working together in groups understand health issues and make decisions about those issues. The theoretical framework draws from a variety of health communication, social influence, and small group theories. Rather than solely emphasizing individual level behavior change, this study recognizes that individuals exist within social groups and that group norms can influence our health behaviors. To better examine the process of group normative influence on a specific health issue, this study employed social network analysis of complete groups. Specifically, the cognitive social structure (CSS) was adapted to examine collective work group norms around a precise health issue. For this study, a single health issue was examined: H1N1 flu prevention. To increase the generalizability of the research to other health choices, two distinct H1N1-related behaviors were studied: intention to get the H1N1 flu vaccination and willingness to stay home from work if sick with the H1N1 flu.

Recently, Fishbein [8,9] updated the theory of reasoned action and the theory of planned behavior into a new integrative model of behavioral prediction (IMBP). The theory of reasoned action (TRA) is a cognitive theory that states that attitudes and subjective norms predict behavioral intentions [10,11]. Attitudes are assessments of negative or positive feelings toward expected outcomes if the behavior is performed. Subjective norms are measured by multiplying normative beliefs for specific relevant others by motivations to comply with those relevant others [12]. To expand the TRA’s applicability beyond solely those behaviors under an individual’s control, Ajzen proposed the addition of perceived behavioral control as a third factor predicting behavioral intention in his theory of planned behavior [12,13]. Perceived behavioral control is similar to Bandura’s concept of self-efficacy [14]; it is the extent to which individuals feel that the ability to perform the behavior is within their influence.

For the IMBP, Fishbein and colleagues [8,9] developed these models further by suggesting that both actual ability level and facilitators and barriers in the environment join behavioral intentions in predicting behavior. Moreover, they broadened the subjective norms concept to a more general conception of social norms to emphasize the importance not only of what referent others expect but also of what people actually do as an important social motivator [15]. Thus, the IMBP highlights attitudes, social norms (both subjective and descriptive), and self-efficacy as the proximal predictors of behavioral intent. It is crucial that each of the constructs included to be specific to the behavior in question.

Several studies have examined adults’ attitudes and intentions about H1N1 flu. Intentions to get the vaccine were typically lower than intentions to follow other CDC recommendations for H1N1 prevention [16]. This discrepancy may be partially attributable to concerns about vaccine safety more generally. Intentions to be vaccinated for H1N1 were strongly positively associated with vaccination behavior for seasonal flu, “suggesting common attitudinal barriers to both vaccines” ([17], p. 5732). Moreover, intentions to get the H1N1 vaccine were predicted by attitudes, subjective norms, perceived benefits, and perceived barriers [18].

Based on the health theories and research described above, several constructs can be identified as likely predictors of behavioral intentions with regards to H1N1. The following hypothesis is postulated:

Hypothesis 1. (a) Attitudes, (b) self-efficacy, (c) subjective norms, and (d) descriptive norms are positively associated with behavioral intentions both to be vaccinated for H1N1 and to stay home from work if sick with H1N1.

Researchers have examined the impact not just of social norms generally but also of norms for specific social groups [3,19,20,21]. According to the theory of normative social behavior (TNSB), both feeling similar to one’s social group and wanting to be like the group moderate the influence of descriptive norms on behavior. When considering their own behavioral choices, people can compare their decisions not only to a general societal norm about health behaviors but also to norms for particular reference groups of which they are a member or that they deem important [22]. Small group research within the social identity perspective suggests possible mechanisms for the development and maintenance of group norms. According to the social identity perspective, members of a group share a social identity. When the identity is salient, group members categorize in a way that emphasizes the difference between their group and other groups, and they particularly emphasize the differences that favor their own group [21]. The group shares an understanding of how a prototypical group member does and should act. Group members gain respect from their peers by acting in accordance with this ideal. Thus, these shared understandings can become both descriptive and injunctive norms of how members do and should act [23]. Such norms can be internalized and have an impact even in the absence of other group members [24]. Much of the research on work group norms examines norms related to working and unrelated to the health domain; in contrast, the current study applies the concepts from social identity theory to norms around a health issue that may not be central to the work environment but is implicated by it.

Hypothesis 2. Individually perceived group norms are positively associated with individual behavioral intentions both to be vaccinated for H1N1 and to stay home from work if sick with H1N1.

In contrast to the importance of motivations to comply for the IMBP, Terry *et al.* suggested that group norms do not act solely through motivation to comply or concerns over social sanctions [21]. Additionally, individuals’ understandings of themselves based on their group membership guide their behavior. Thus, Terry and Hogg hypothesized and found that attitudes that are congruent with perceived group norms are most predictive of behavioral intentions for people who have strong group identities [20]. Which group identity individuals perceive as salient is crucial. Activating a particular group prototype not only makes associated attitudes more accessible, but it also makes them normative by highlighting the social group consequences of behavior [21]. Thus, both group norms and the salience of those norms are important in determining behavior. This literature suggests two possible moderators of individuals’ perceptions of group norms on behavioral intentions.

Hypothesis 3. Motivations to comply moderate the relationship between group norms and individuals’ behavioral intentions, such that for those who are more motivated to comply with group members’ wishes, group norms will be more strongly associated with behavioral intentions both to be vaccinated for H1N1 and to stay home from work if sick with H1N1.

Hypothesis 4. Group identification moderates the relationships between group norms and individuals’ behavioral intentions, such that for those who identify more strongly with the group, group norms will be more strongly associated with behavioral intentions both to be vaccinated for H1N1 and to stay home from work if sick with H1N1.

The first four hypotheses are based on existing social science theories commonly applied to health communication. However, they share a major constraint in that each is typically examined at the individual level only. Although they theorize about the broader social environment, the influence of that environment is commonly assessed as perceived by specific individuals. Social network analytic techniques that leverage complete groups can help us to answer the call for more ecological approaches to health and to add insight into how individuals make health decisions.

In previous efforts to examine the role of social structure in influencing health decisions, researchers have used social network analysis [25]. Rogers suggested that innovations and new ideas are diffused through social networks [26]. Within these networks, people learn appropriate behaviors as they talk about how messages are received [5,6,27,28]. Christakis and Fowler have used social network analysis to examine how social networks relate to health status [29,30,31]. In a longitudinal analysis of the Framingham Heart Study data, they found that people’s chance of becoming obese increased if they were directly connected to another individual who became obese during the study interval [29]. Likewise, smoking cessation is more likely if others in the social network have ceased smoking [30]. Based on their findings, Christakis and Fowler speculated that social norms could be implicated as a potential reason why social networks are so important [31]. With respect to vaccination behavior, parental choices to vaccinate their children are largely influenced by whether their social network contacts have vaccinated or refused to vaccinate their children [32]. Increasingly, scholars have called for stochastic network analytic techniques that incorporate statistical tests of hypotheses and examine change over time [33,34]. Such techniques can move beyond descriptive social network analysis to advance the field of public health by accounting for the endogeneity of network data. An alternative method that likewise allows hypothesis testing and leverages a social network perspective is to gather data from multiple distinct networks. This study uses such an approach by employing cognitive social structures and examining complete work groups.

Krackhardt introduced the concept of a cognitive social structure as a means to explore how people perceive their social interactions [35]. As compared with traditional network analysis, a cognitive social structure analysis asks each group member about the interactions among each other pair of group members [35]. Specifically, each member of a complete group is asked about both their communication with other group members and about their perceptions of the communication of every other pair in the group. This leads to the creation of a layered network in which each layer, or slice, is an individual’s perception of the entire network. For a group with N participants, a traditional network analysis would include the N × N interactions among the people. In contrast, a cognitive social structure is N × N × N because it includes each individual’s cognitions about the interactions of each other pair of individuals in the network. Given its three-dimensional nature, a cognitive social structure can be collapsed into multiple types of two-dimensional networks. First, a slice is the response of a single individual, or that person’s perception of the complete network. Second, a consensus structure is the matrix that shows what the group as a whole deems to be the interactions among each possible pair.

Such a layered network approach may provide a more complete picture of group social norms than traditionally measured individual level norms, and thus may allow insight into the social influence process for groups. However, to examine this possibility, changes to the traditional cognitive social structure must be made. Instead of simply examining a communication relation, the relation examined must be a normative one. Thus, in this study, participants were asked to report the perceived support for specific behaviors by each other pair in the group. This allows for examination of each individual participant’s perceptions of the group norms, but through the use of the consensus structure, it also allows for the examination of the collective perception of the group about appropriate behaviors. Using social network analysis, the final set of hypotheses uses the CSS to move to a higher level of analysis. Rather than solely focusing on individual level predictors or even individual conceptions of group social norms, the actual norms about H1N1 flu prevention held by the complete group are expected to have an impact on behavioral intentions.

Hypothesis 5. Controlling for individual level predictors, collective group norms as measured by the CSS consensus structure will be associated with behavioral intentions both to be vaccinated for H1N1 and to stay home from work if sick with H1N1.

Hypothesis 6. Controlling for individual level predictors, consistency of collective group norms as indicated by the standard deviation of the CSS consensus structure will moderate the impact of individually perceived group norms on behavioral intentions to be vaccinated for H1N1 and to stay home from work if sick with H1N1.

## 2. Methods

To explore how social norms are understood in small group contexts, a network survey was administered online to groups of adults working together in organizational settings. For this study, the normative behaviors examined related to prevention of the Novel 2009 H1N1 Flu.

### 2.1. Participants

The study population consisted of adults who worked together in California. A work group was operationalized as a group of co-workers at the same organization working in the same physical location. Physical proximity was required to ensure that group members had the possibility of interacting and communicating with each other in both work-related and non-work-related ways. Additionally, work groups had to have defined boundaries that distinguished work group members from other employees who were not members of the same work group. Recruitment was a multi-step process in which organizations were first approached to participate and asked to identify a single work group of approximately seven to ten people. To be eligible, work groups needed to have worked together consistently from fall 2009 when H1N1 became prevalent. From February to May 2010, 83 organizations were contacted to request their participation in the study. Of those contacted, 20 organizations (24%) were ineligible. Ultimately, twenty organizations (32% of those eligible) agreed to participate. Two groups worked at public, nine at non-profit, and nine at for-profit institutions. Organizations were classified as belonging to one of five broad categories based on the type of work performed: health/social service (30%), education (15%), financial/legal services (25%), arts/entertainment/technology (20%), and those that did not fit into the other four categories (10%). Although some organizations included health care professionals, none of the organizations required their employees to be vaccinated for H1N1 flu.

Next, each group member was asked to provide informed consent. All subjects gave their informed consent for inclusion before they participated in the study. The study was conducted in accordance with the Declaration of Helsinki, and the protocol was approved by the University of Southern California University Park Institutional Review Board (#UP-09-00416). The multi-stage recruitment process led to a high response rate among individuals (94%, 152 respondents). Thirty-nine percent of respondents were male, and 57% were female. Participants’ ages ranged from 21 to 67 years old, with a median age of 32. Forty-six percent of participants were white, 9% were black, 16% were Hispanic, 20% were Asian or Pacific Islander, and 5% were of another race or ethnicity.

### 2.2. Survey

Two specific H1N1-related behaviors were studied: intention to get the H1N1 flu vaccination and willingness to stay home from work if sick with the H1N1 flu. The social cognitive variables were assessed separately for each behavior. The survey was conducted using an online software program that piped group members’ names into the survey.

To measure behavioral intentions, survey respondents were asked how likely they were to get the H1N1 vaccine and how long they would be willing to stay home from work if they were to become sick (measured in number of days).

Following Fishbein [10], attitudes toward H1N1 vaccinations and toward staying home while sick were assessed using four six-point semantic differentials anchored by favorable/unfavorable, risky/safe, bad/good, and responsible/irresponsible. The responses were averaged separately for attitudes toward H1N1 flu vaccinations (Cronbach’s α = 0.90) and toward staying home while sick from H1N1 flu (Cronbach’s α = 0.78).

Self-efficacy was assessed for each behavior separately through the one-item measures: “I feel able to get an H1N1 swine flu vaccination” and “I feel able to stay home from work if sick with H1N1 swine flu” with 7-point Likert scales ranging from 1 = strongly disagree to 7 = strongly agree. This choice follows IMBP inclusion of self-efficacy and Armitage and Conner’s operational definition of self-efficacy as “confidence in one’s own ability to carry out a particular behavior” [36] (p. 479), rather than the related construct, perceived behavioral control.

Subjective norms were measured by assessing both normative beliefs and motivation to comply [27,28]. Specifically, normative beliefs were measured for relevant others including parents, doctors, and other friends. Each respondent was asked how much those people wanted them to be vaccinated for H1N1 swine flu (Cronbach’s α = 0.90) and how much those people would want them to stay home if they became sick with H1N1 swine flu (Cronbach’s α = 0.85). Although the TRA strongly suggests the importance of matching attitudes, subjective norms, and behavioral intentions to specific behaviors in context [10], motivation to comply is often measured more generally. For example, Boer and Mashamba asked respondents to indicate the extent to which they agreed with the following, “I care about the opinions of my friends” [37]. In this survey, motivations to comply were measured with behavioral specificity for each of the behaviors under study. Motivations to comply were measured as how much the opinion of each group member mattered to the respondent, separately for vaccination (Cronbach’s α = 0.85) and staying home (Cronbach’s α = 0.87). Response options for both types of questions were 10-point scales. The order of the normative belief and motivations to comply questions were randomly counterbalanced for the different work groups.

Following Rimal and Real [3], respondents were asked to estimate the percentage of people their age who were vaccinated for H1N1 swine flu or would stay home from work if they were sick with H1N1 swine flu as a measure of descriptive norms.

To fully measure work group identification as recommended by Olkkonen and Lipponen, scales measuring both cognitive and affective components were included on the survey [38]. The eight item Affective Commitment Scale [39] included items such as “This work group has a great deal of personal meaning for me” (Cronbach’s α = 0.85). The cognitive components of work group identification were measured using Mael and Ashforth’s six item organizational identification scale [40], with an example item being “When I talk about my work group, I usually say ‘we’ rather than ‘they’” (Cronbach’s α = 0.76). Both were measured with 7-point Likert scales ranging from 1 = strongly disagree to 7 = strongly agree.

The cognitive social structure (CSS) for each group was adapted from Krackhardt’s original conception [35]. Rather than ask participants who knew who else in the group, participants were asked for each pair of members in their group how supportive of H1N1 vaccination a conversation between them would be (see Figure 1). The responses of each individual were used to generate that individual’s CSS slice. In other words, these responses were the individual’s perception of how supportive all dyads in the work group are of H1N1 vaccination. The locally aggregated structure (LAS) indicates what was reported by the individual pairs about their support for H1N1 vaccination. The layering of all of the individual slices from a particular work group formed the CSS in support of H1N1 vaccination for that group. For each work group, the CSS consensus structure was calculated by taking the mean of the cells for each member’s slice. Thus, this adaptation of the CSS includes three ways of viewing group social norm data: (1) slices—the individual’s perceptions of pair support, (2) LAS—the perceptions of pair support by just the two partners involved, and (3) consensus structures—the average group perception of the pair support for vaccination. Because the focus of this study is on individual’s perceptions of their group norms and the collective perception of the group norms, only the individual CSS slices and the group CSS consensus structures were used for analysis.

For interval-level data such as that used here, network density indicates the average tie strength across all possible ties [41]. In other words, the density of the consensus structure (the overall average perceived support by all work group members of each dyad in the group) represents the overall group social norms, or the level of support for vaccination, indicated by the group collectively. In addition to the overall level of support, it is important to also consider the consistency of that support across the pairs of group members, as H6 hypothesized that this would moderate the effect of individual CSS slices on behavioral intentions. The standard deviation can be calculated as a measure of the “separation” of different group members [42]. High standard deviation of the CSS consensus structure indicates low levels of group agreement about support for a health issue such as vaccination.

### 2.3. Analysis

Analysis was conducted using social network analysis with UCINET and hierarchical linear modeling (HLM6). UCINET was used for network data preparation by stacking the CSS slices to compute the consensus structures. The densities of each individual’s slice of the CSS (each individual’s perception of the average support for vaccination and staying home) were calculated as individual level predictors. Additionally, the overall density and standard deviation of the group’s CSS consensus structure were calculated as group level variables.

**Figure 1:** Cognitive social structure components.

All hypotheses testing the association between variables were examined using two level hierarchical linear modeling (HLM) and hierarchical generalized linear modeling (HGLM) to control for interdependencies among group members [42,43,44]. For each dependent variable, a series of analytical steps were taken. First, the null or baseline model was estimated to calculate the intraclass correlation coefficient (ICC, the percentage of variance in the dependent variable that is attributable to group membership). Second, after the null, unconditional model was estimated, hierarchical linear models were run with level-1 (individual) predictors added. In the third step, level-2 (group) predictors were added to the model. Depending on the specific hypothesis being tested, the effects of the group level predictors were estimated for the individual level intercepts or for the individual level slopes.

## 3. Results

The individual means and the standard deviations for each are presented in Table 1. There are three different conceptions of social norms included: (1) subjective norms from the IMBP which are the summed product of normative beliefs and motivations to comply with, (2) descriptive norms which are the percentage of people that respondents think engage in the specified behaviors, and (3) cognitive social structure (CSS) slices which are the individuals’ perceptions of the norms of the group as a unit. As can be seen in the table, there are generally higher levels of support for staying home from work if sick with H1N1 than for becoming vaccinated.

The intention to stay home from work if sick with H1N1, as measured by days that the respondent would be willing to stay home, was highly skewed. Therefore, it was categorized into three groups: those willing to stay home at most five days, between six and ten days, and more than ten days. The assumption of proportional odds necessary for ordinal HGLM models was violated, so nominal, multinomial HGLM models were estimated for the intention to stay home if sick using restricted penalized quasi-likelihood estimation [44,45,46].

**Table 1:** Individual level descriptive statistics about H1N1 flu prevention.

	H1N1 Vaccination		Staying Home from Work if Sick	
	Mean	SD	Mean	SD
Attitudes ^a^	4.4	1.6	6.6	0.8
Self-efficacy ^a^	5.2	1.8	6.3	1.2
Subjective norms ^b^	18.7	21.7	62.9	31.0
Motivations to comply ^c^	3.7	2.7	6.5	3.0
Descriptive norms ^d^	30.2	16.8	75.8	21.9
CSS slice group norms ^e^	3.1	0.6	3.9	0.3
Behavioral intentions ^f^	3.2	2.5	9.7	12.1

^a^ Scale ranges from 1 to 7; ^b^ Scale ranges from 1 to 100; ^c^ Scale ranges from 1 to 10; ^d^ Response is a percentage; ^e^ Scale ranges from 1 to 4; ^f^ For vaccination, scale ranges from 1 to 10, and for staying home, the number of days willing to stay home if sick with H1N1.

The first hypothesis suggested that attitudes (H1a), self-efficacy (H1b), subjective norms (H1c), and descriptive norms (H1d) would all be positively associated with behavioral intentions (see Figure 2 for a figure summarizing hypotheses and results). Attitudes (γ = 0.66, *t* (135) = 4.47, *p* < 0.001) and subjective norms (γ = 0.03, *t* (135) = 2.52, *p* < 0.05) were significantly associated with H1N1 vaccination intentions (see Table 2 for a summary of the HLM models of vaccination intentions). In contrast, while controlling for the participant’s gender, only self-efficacy significantly predicted intentions to stay home if sick (see Table 3 for a summary of the HGLM models of intentions to stay home). Increasing levels of self-efficacy were significantly related to increased likelihood to stay home for six to ten days (OR: 2.43, CI: 1.15–5.15, *p* < 0.05) and marginally related to increased likelihood to stay home for more than ten days (OR: 1.90, CI: 0.94–3.88, *p* = 0.075).

While controlling for individual level predictors, Model Vaccination 2 (see Table 2) adds in the individually perceived group norms of the cognitive social structure and hypothesized individual-level moderators. Specifically, H2 was that the cognitive social structure would also relate to behavioral intentions. The fixed effect of CSS slice density on behavioral intentions was not statistically significant. H2 was not supported for vaccination. H3 and H4 examined variables that might moderate the influence of group norms on behavioral intentions: motivations to comply and work group identification. Motivations to comply significantly moderated the impact of perceived group norms on behavioral intentions to become vaccinated (γ = 0.07, *t* (134) = 2.9, *p* < 0.01). Likewise, the cognitive aspect of work group identification also significantly moderated the impact of perceived group norms on intentions (γ = 0.28, *t* (134) = 2.4, *p* < 0.05). However, the affective measure of workgroup identification was not a moderator. Thus, H3 (motivations to comply) was strongly supported for intention to get the H1N1 vaccination; H4 (work group identification) was supported for the cognitive aspect only.

As with intentions to vaccinate, to test H2 for intentions to stay home if sick with H1N1, an HGLM model was similarly estimated controlling for the two predictors previously found to be significant, gender and self-efficacy. The odds ratio of CSS slice density for staying home was not significantly related to behavioral intentions either for willingness to stay home six to ten days (see Model Home 2: OR: 1.60, CI: 0.23–11.1, *p* = .63) or for willingness to stay home more than ten days (OR: 0.85, CI: 0.12–6.15, *p* = .87) compared to willingness to stay home five days or fewer. H2 was not supported for intention to stay home from work if sick. Simultaneously, the interaction hypotheses (H3 and H4) were also tested for willingness to stay home if sick with H1N1. Controlling for gender and for self-efficacy, none of the interaction effects of group norms on behavioral intentions were significant. Unlike for vaccination, for behavioral intentions to stay home if sick with H1N1, H3 and H4 were not supported.

**Figure 2:** Summary of results.

**Table 2:** Summary of hierarchical linear modeling (HLM) results for predictors of H1N1 vaccination intention.

Fixed Effects (Predictors)	Model Vaccination 1	Model Vaccination 2	Model Vaccination 3
Intercept	3.18 **	3.22 **	3.20 **
Attitudes	0.66 **	0.62 **	0.60 **
Self-efficacy	0.00	-	-
Subjective norms	0.03 *	-	-
Descriptive norms	0.01	-	-
CSS slice group norms	-	−0.05	0.45 *
Motivations to comply x CSS slice group norms	-	0.07 *	0.07 **
Cognitive work group identification x CSS slice group norms	-	0.28 *	-
Affective work group identification x CSS slice group norms	-	−0.16	-
CSS consensus group norms	-	-	1.59 *
CSS consensus group norm separation x CSS slice group norms	-	-	−6.40 **
*R*^2^ (Additional level-1 variance explained compared to null model)	23.5%	21.5%	25.5%
*R*^2^ (Additional level-2 variance explained compared to null model)	-	-	7.6%
Random Effects	Deviance	Variance	χ*^2^* (*df*)
Model Vaccination 1: Intercept, *u*_0_	516.692	0.649	36.5 (19) **
Level 1 variance, *r_ij_*	-	4.057	
Model Vaccination 2: Intercept *u_0_*	525.874	0.734	38.4 (19) **
Level 1 variance, *r_ij_*	-	4.093	
Model Vaccination 3: Intercept, *u*_0_	520.307	0.482	30.7 (18) *
Level 1 variance, *r_ij_*	-	4.167	-

* *p* < 0.05; ** *p* < 0.01.

**Table 3:** Summary of hierarchical generalized linear modeling (HGLM) results for predictors of intention to stay home if sick.

Fixed Effects (Predictors)	Willing to Stay Home 6–10 days ^a^		Willing to Stay Home >10 days ^a^	
	Odds ratio	Confidence Interval	Odds ratio	Confidence Interval
Model Home 1				
Intercept	0.54	(0.27, 1.10)	0.43 *	(0.23, 0.79)
Gender (reference is male)	1.16	(0.39, 3.42)	0.23 *	(0.07, 0.76)
Attitudes	1.11	(0.53, 2.35)	1.89	(0.76, 4.70)
Self-efficacy	2.43 *	(1.15, 5.15)	1.90	(0.94, 3.88)
Subjective norms	1.01	(0.99, 1.02)	1.00	(0.99, 1.03)
Descriptive norms	1.01	(0.99, 1.03)	1.02	(0.99, 1.05)
Model Home 2				
Intercept	0.63	(0.35, 1.12)	0.44 **	(0.25, 0.77)
Gender (reference is male)	1.11	(0.41, 3.03)	0.31 *	(0.11, 0.91)
Self-efficacy	1.32	(0.89, 1.94)	2.25 *	(1.17, 4.33)
CSS slice group norms	1.60	(0.23, 11.06)	0.85	(0.12, 6.15)
Motivations to comply x CSS slice group norms	1.00	(0.97, 1.05)	1.01	(0.97, 1.06)
Cognitive work group identification x CSS slice group norms	0.97	(0.75, 1.24)	0.98	(0.75, 1.27)
Affective work group identification x CSS slice group norms	1.21	(0.95, 1.54)	1.19	(0.92, 1.55)
Model Home 3				
Intercept	0.60	(0.34, 1.08)	0.37 **	(0.20, 0.69)
Gender (reference is male)	1.21	(0.46, 3.22)	0.32 *	(0.11, 0.93)
Self-efficacy	1.33	(0.91,1.96)	2.81 **	(1.36, 5.78)
CSS slice group norms	3.83	(0.32, 45.30)	3.27	(0.18, 59.71)
CSS consensus group norms	1.05	(0.01, 80.29)	96.3 *	(1.16, 7996)
CSS consensus group norm separation x CSS slice group norms	0.00	(0,4.9 E9)	0.00	(0,1.5 E11)

^a^ Reference group is those willing to stay home a maximum of 5 days; * *p* < 0.05; ** *p* < 0.01.

The final hypotheses, H5 and H6, incorporate group level predictors of behavioral intentions. Specifically, H5 hypothesized that while controlling for individual level predictors, the group level density of the consensus structure of the CSS would both have a direct effect on behavioral intentions and would moderate the impact of individually perceived group norms on behavioral intentions. H6 hypothesized that the consistency of this consensus structure (as measured by the standard deviation) would also have a cross-level interaction effect by moderating the impact of individually perceived group norms on behavioral intentions. H5 was supported. The group level CSS consensus structure density is positively associated with behavioral intentions, even when controlling for the individual slice density (see Model Vaccination 3: γ = 1.59, *t* (18) = 2.7, *p* < 0.05). It is interesting to note that in this model with group level and interaction effects included, the individually perceived group norms are also statistically significant as was originally hypothesized in H2 (γ = 0.45, *t* (135) = 2.0, *p* < 0.05). Similarly, H6 was supported. The more consistent (lower standard deviation) the CSS consensus structure was, the stronger the relationship between the individual CSS slice density and behavioral intentions to get vaccinated (γ = −6.40, *t* (135) = −2.9, *p* < 0.01). Model Vaccination 3 shows the final model for H1N1 vaccination intention. With the direct and interaction effects included, this model explains 26% more of the individual level variance and 8% more of the group level variance than the unconditional model does.

Hypotheses 5 and 6 were also tested for intention to stay home if sick with H1N1. As for H1N1 vaccination intention, H5 was supported. While controlling for individual level predictors of gender, self-efficacy, and individual CSS slice density, the group level CSS consensus structure density was significantly positively associated with willingness to stay home more than ten days relative to those willing to stay home five days or fewer (see Model Home 3: OR: 96.3, CI: 1.16–7966, *p* < 0.05). The very large odds ratio and confidence interval suggest a lack of precision due to small cell sample size, so H5 received tentative support. However, H6 was not supported. The consistency of group support did not moderate the impact of the individually perceived group norms on behavioral intentions to stay home.

## 4. Discussion

This study examined multiple influences on health-related intentions for H1N1 flu prevention behaviors using an adapted cognitive social structure and social network analysis. In the following paragraphs, I detail implications for H1N1 flu prevention, public health communication theory, and the conceptualization and operationalization of group norms. As hypothesized, individuals’ attitudes, self-efficacy, and subjective norms all related to behavioral intentions for at least one of the H1N1 health behaviors under study. While controlling for individual level predictors, the groups’ consensus about the health-related social norms of the whole group had an additional impact on behavioral intentions for both H1N1 vaccination and willingness to stay home from work if sick. For members of work groups in which pairs were perceived to agree in their support for H1N1 vaccination, the effect of individually perceived group norms on behavioral intentions was stronger than for groups with less agreement.

For H1N1 vaccination, motivation to comply had a significant interaction effect. In other words, for people who were strongly motivated to comply with their co-workers, individually perceived group norms had a stronger relationship with behavioral intentions for this health behavior. Likewise, the cognitive component of workgroup identification had a similar moderating effect. However, neither was significant for willingness to stay home from work if sick with H1N1. Terry *et al.*’s research indicated that motivations to comply would not be as important as work group identification in moderating the impact of group norms [20]. The results found here suggest that modifications to this premise are necessary. Perhaps work group identification is more important than motivation to comply only when the behavior in question is prototypical of the group or when directly related to the group’s work product. Health behaviors (both related to H1N1 but also more generally) are unlikely to be a strong defining component of how a work groups sees themselves. Thus, for health behaviors, work group identification may not be as important as motivations to comply. In the health realm, the more proximal motivations to comply and the salience of the health behavior to the work environment may be the most important theoretical constructs to moderate the impact of group norms on individuals’ behavior.

The cognitive social structure (CSS) included both individual slices of the perceived group norms and a consensus structure that averaged those slices for the whole group. In this way, it included both individually perceived group norms and the collective norms of the complete group. The individual perceptions of the group norms about H1N1 vaccination as indicated by the CSS slice density were positively associated with behavioral intentions toward H1N1 vaccination. When individuals perceived pairs of group members to be supportive of vaccination, they were more likely to report intending to get the vaccine themselves. However, the individual CSS slices were not predictive of willingness to stay home if sick with H1N1.

The group CSS consensus structure leveraged responses from the entire group to measure the collective group norms. This CSS consensus structure was predictive of behavioral intentions for both the H1N1 vaccination intention and willingness to stay home from work if sick with H1N1. Even after accounting for individuals’ perceptions of the group norms, the actual group consensus about the normative support for both behaviors had a direct impact on work group members’ intentions for both health behaviors. In work groups with high levels of support for vaccination or staying home from work, members were more likely to intend to engage in those behaviors, respectively. The consistency of the group CSS consensus structures, shown by low standard deviations, moderated the impact of individually perceived group norms on behavioral intentions for H1N1 vaccination. For members of work groups in which pairs were perceived to agree in their support for H1N1 vaccination, the effect of individually perceived group norms on behavioral intentions was stronger than for groups with less agreement.

The findings of this study have theoretical and methodological implications for both the study of health behavior and the impact of group norms on behavior more generally. To date, much research in public health has focused on the individual level predictors of behavior. By combining the constructs with the most predictive validity from a variety of health communication theories, the integrative model of behavioral prediction (IMBP) has become a strong individual-level theory [8,9]. However, the findings here suggest that individual level predictors are not necessarily the most important. In fact, only group level social norms as measured by the CSS were significantly predictive of behavioral intentions for both H1N1 flu prevention behaviors in every model run. Therefore, higher levels of analysis must be considered to advance theorizing on health behavior choices. Taken together, the group level effects highlight the importance of assessing entire groups and explicitly incorporating the social environment into understandings of health behaviors. Individually perceived norms alone cannot fully account for individuals’ disease prevention choices. Instead, group level effects are also important, even in cases where the individual perceptions of such group norms may not be predictive of behavioral intentions. The incorporation of CSS into public health communication was supported. The finding that group level social norms are significant for both of H1N1 behaviors provides greater support for the inclusion of the CSS in future work than would study of only a single behavior. This study adds to the literature on group norms by highlighting the importance of collective, or group level, understandings of group social norms. The social context has implications for health choices beyond the way in which that context is perceived by individuals. Thus, an ecological model of health communication with accompanying operationalization and social network analytic techniques is essential for future theorizing about health behaviors. Rather than solely focusing on predicting individual behavior, it must be recognized that individuals exist within social groups, and those groups reside in a wider socio-cultural context.

The methods for this study suggest several innovations that could be incorporated into future research both in public health and in small group research. CSS uses social network analysis to elicit information about social groups. Rather than relying on a simple matrix of who talks to or is influenced by whom, the CSS calls for a further level of data by incorporating each individuals’ understanding of each other pair in turn. Asking about every possible pair in the work group is time consuming, but it provides a more complete understanding of the group interactions than can be obtained by simply asking each individual to report on each other individual. The interactive nature of group social norms is explicitly incorporated into the CSS questions and structure.

The consistency of the group’s collective social norms as indicated by the standard deviation of the CSS consensus structure adds further value to the CSS. Not only can the CSS measure the group’s collective norms, but it also measures the agreement around these norms. This consistency measure provides information different from that obtained by asking individual group members to provide their attitudes and then calculating the standard deviation to determine the agreement across the group. Instead, the standard deviation of the CSS consensus structure incorporates the extent to which the pairs are understood by the group to agree with each other. Again, this group level understanding is an important contribution of the CSS.

In summary, this revised cognitive social structure is a step towards better understanding group social norms and interactions both as applied to health behaviors and more generally. The social environment is important in its potential influence on individual choices. The ability to measure the way in which this social context can influence health is crucial to being able to better theorize about health behaviors. However, this study is by no means the final step towards developing better methods of examining social influences and group social norms. Further work must be done to explore how membership in multiple and possibly overlapping social groups influences health behaviors. Additionally, more constructs should be created that provide good measurements of the overall cultural context, and not just of the people who are closest to the study participants.

### Limitations and Implications for Future Research

Some of the limitations for this study stem from the survey design. The survey was quite long, particularly for people in large work groups. With every additional person in a work group, each network question increased by one item, and each CSS question increased by the same number of items as there were work group members. To limit survey length, some of the constructs were measured with single item scales, rather than longer multi-item scales that may have been more valid. Respondents were able to complete the survey in multiple sessions if they preferred, but most (90.8%) completed it in a single day. Given the length of the survey and that all behavioral questions were asked both for H1N1 vaccination and for staying home from work if sick with H1N1, it is possible that participants suffered from survey fatigue. To account for this, the behavioral questions were counter-balanced by group in their order of presentation. During statistical analysis, there were no order effects, a fact that suggests that survey fatigue played a limited role.

Work group size presents a trade-off. Smaller work groups allow participants to better think through their entire group when reporting. However, small work groups also lead to smaller samples and decreased precision in estimating statistics. In particular, only 36 participants (23%) reported being willing to stay home if sick for greater than 10 days. The small overall numbers in this category and even smaller numbers when nested within groups led to a lack of precision in the odds ratio for CSS consensus group norms. Although the odds were significantly greater than 1, the large point estimate and its confidence interval do not provide useful information about the precise association of group norms with staying home from work if sick.

Use of the CSS relies on data collection from a complete group. Recruitment and informed consent processes are both considerably more complicated when gathering data about complete groups than when asking individuals to complete surveys. Additionally, administration of the CSS is quite time-intensive. With every additional person in a work group, each CSS question increased by the same number of items as there were work group members. However, the collective group norms measured in this manner have an impact on behavioral intentions above and beyond the impact of how those group norms are perceived by individual group members. This makes it important to gather data from each group member. If the design for a particular study does not allow for survey distribution to groups, then ego networks that simply use individual slices of the CSS could be substituted for the collective group norms in this analysis. However, these slices can only capture individuals’ perceptions of the groups’ norms and interactions, not the group level perceptions of norms. Therefore, they are not as strong a means of examining the social context as the complete CSS. Future surveys employing CSS structures would benefit from only including a single behavior to limit overall survey length. The use of the CSS is most appropriate to environments in which clear small groups are identifiable by group members.

This study followed the work of Fishbein and Ajzen in examining behavioral intentions as a primary outcome [11]. Although shown to be a strong predictor of actual behaviors, behavioral intentions are not of primary importance theoretically. Instead, they are used as a proximal indicator of behavior. As noted by the integrative model for behavioral prediction (IMBP), the path from behavioral intentions to actual behaviors may be influenced by individuals’ actual skills or abilities and any barriers from the environment [8,9]. For the present study, the H1N1 vaccine shortage made obtaining a vaccine difficult. Moreover, actual behaviors in staying home from work were only relevant for those people who actually contracted the H1N1 flu. Thus, for both of these behaviors, intentions were chosen as a better way to examine the influence of the social environment. However, future studies should not automatically explore behavioral intentions.

## 5. Conclusions

The current study found that group social norms as assessed through social network analysis of complete work groups are important predictors of individual behavioral intentions for H1N1 flu prevention. Although individual predictors and perceptions of social norms were associated with behavioral intentions, much action took place at the group level. Over and above any individual level effects, social norms as understood by the entire work group were consistently strongly related to individuals’ behavioral choices. Though this study only examined two health behaviors, the findings have generalizability beyond H1N1 flu prevention. The two different types of H1N1 behaviors studied were chosen because they differed from each other significantly. For H1N1 flu, individuals both can choose whether or not to be vaccinated (a relatively private choice that primarily impacts their own health) and whether to stay home from work if they become sick (a public choice that can also impact the health of others). These behaviors resonate with similar behaviors in the health field. As discussed above, choices around H1N1 vaccination have much in common with decisions to receive other vaccines [17]. Likewise, the CDC commonly recommends that people stay home from work whenever they are contagious. People’s choices to comply with such instructions from authorities, including the choice to shelter at home, are known to be associated with beliefs in the preparedness of the local health care system and perceived response efficacy of complying with government instructions [47]. For both of these behaviors, work group social norms should also be considered in future public efforts for prevention. Campaigns should be structured around the group norms that match the situation and salient group identity. Increasingly, organizations that provide health insurance to their employees are encouraging programs that promote health and prevention of disease. Better understanding of the work environment and the shared norms of co-workers will be crucial to the success of such health initiatives. Programs that highlight the impact of choices to vaccinate or other health behaviors on colleagues may prove particularly useful. If employers wish to encourage healthy choices for behaviors that are seen as more private, then stronger messaging and work place incentives may be necessary. For example, vaccination should be reframed as a preventive measure that can improve immunity for the entire office setting. By tying vaccination to a group norm, it may have a stronger influence on behavior than when seen as solely an individual or private choice.

In addition to these implications for public health interventions, these data underscore the importance of using existing, complete groups to study the group social influence process. By looking not just at the individual level but also at the group social context, a greater understanding of health issues, such as flu prevention, can be achieved. Integrating group level conceptions of social norms into health communication theories will allow a more complete and nuanced understanding of health behaviors. This study highlights the fact that individuals do not live in vacuums but rather are inextricably part of various social groups, each of which may have a distinct impact on their health-related choices.
